RETRACTED

# Relationship between Volleyball Sports Nutrition Food and Sports Athletes' Training and Physical Health Based on Medical Image Recognition

**DOI:** 10.1155/2021/2214359

**Published:** 2021-12-10

**Authors:** Jian Liu

**Affiliations:** Institute of Physical Education, East China University of Technology, Nanchang, 330013 Jiangxi, China

## Abstract

As we all know, the dietary nutrition of athletes has a great influence on physical condition and exercise ability. A good diet pattern is the basis of a reasonable diet for athletes. It helps to improve the function and physical state of athletes. This article is aimed at studying the impact of nutritious food on athletes' training and physical health. This article proposes the relevant technology of medical image recognition, which is used to study the relationship between nutritious food and the health of volleyball players and athletes, and proposes methods such as weighing method, meal review method, and measurement method, and the purpose is to exercise nutritional research and provide new ideas and methods. In addition, 200 female volleyball players were randomly selected for comparative analysis. The experimental results in this paper show that the energy intake and energy consumption of the female intervention group maintained a balance after the intervention, and there was a significant change in the negative balance state before the intervention. The energy consumption changed from −158.2 ± 156.2 to −157.2 ± 129.6. The number of athletes whose weight is close to the ideal range has increased from 44.8% to 48.5%.

## 1. Introduction

### 1.1. Background

At present, medical images are widely used in clinical detection and have become an important means for doctors to assist in diagnosis, disease evaluation, and treatment. In recent decades, due to the rapid development of computer technology, the imaging speed and resolution of medical imaging equipment have been greatly improved, and the medical image data has also shown a blowout growth. The improvement of athletes' performance should be attributed to reasonable sports training. Of course, the basis of all this is that athletes have a healthy body. As we all know, athletes' diet should be strictly controlled. Due to the particularity of the industry, they need to supplement appropriate nutrition, how much and what nutrition to supplement, all of which are required. Therefore, the research on sports nutritional food is very necessary. This paper will study the relationship between sports nutritional food and athletes' training and health.

### 1.2. Significance

Material and energy metabolisms are the basis of the functional activities of various tissues and organs. On the whole, the energy consumed by the body's exercise is obtained from energy substances such as sugar, fat, and protein through digestion and absorption. Therefore, applying the laws of substance and energy metabolism during exercise, arranging a reasonable diet, and balanced nutrition are not only necessary for weight and body composition control but also help athletes to exert training effects, improve athletic ability, and promote physical recovery after exercise. Therefore, how to arrange diet and training during weight control so that athletes can maintain good physical quality and competitive state and successfully complete the competition task. This has become an urgent issue in war preparation. Volleyball players have outstanding physical quality, great development potential, and high cultural quality; however, insufficient training and insufficient attention to special physical training. At present, the special physical quality of college women's volleyball players is also easy to be ignored. Therefore, it is of great theoretical significance and practical value to pay attention to the diet and nutrition of volleyball players and the cultivation of athletes' physical quality.

RETRACTED

### 1.3. Related Work

Volleyball is a physical exercise that combines short bursts of height, speed, and strength with short intervals. Hui investigated and field experiment on nutrition intervention for football players and put forward and proved the practical basis and empirical effect of nutrition supplementation for football players. The purpose is to provide an effective basis for supporting the nutritional supplementation of football players through targeted case studies [1]. Waller aims to update Australian athletes' knowledge of the use of supplements in national sports agencies. The authors used an online questionnaire to conduct a cross-sectional survey to assess the effects of age, sport type, and scholarship type on supplement use. The results of this study show that the use of supplements is high, and for the first time shows the impact of social media, especially on young athletes. There are opportunities to optimize how athletes are informed about supplement use and organization and supplement policy [2]. Wang et al. proposed that most of the current medical images are collected in the presence of interference, such as light, occlusion, and other neglected interferences. For multiresolution images, the recognition rate is low when the colors are distorted. The author proposes a new fuzzy clustering recognition algorithm for multiresolution medical images. Experimental results show that this method has a higher recognition rate (accuracy rate of 90.46%, sensitivity of 97.89%) and stronger anti-interference ability than existing methods [3]. Wan et al. researched the problem of insufficient detail retention in sparse representation (SR) multimodal medical image fusion (MMIF) and proposed a MMIF method based on density peak clustering and convolutional sparse representation (CSR-DPC). First, the base layer is obtained through the average filter according to the registered input image, and the original image is subtracted from the base layer to obtain the detail layer. Experiments show that, compared with the two most advanced multiscale transformation methods and five SR methods, the proposed method (CSR-DPC) is superior to other methods in terms of image details, visual quality, and objective evaluation. Contribute to clinical diagnosis and adjuvant treatment [4]. Kaya et al. aims to investigate the relationship between nutritional habits, body mass index, and academic performance of college students. The method used is to conduct a questionnaire survey of volunteer students and attach an informed consent form to determine sociodemographic characteristics, eating habits, and body mass index. The conclusion is that the eating habits of students are related to academic performance. Special attention should be paid to nutrition to cultivate a healthy, productive, and successful generation during adolescence. During this period, the development will continue and the habits developed may continue in adulthood [5]. Surdu et al. investigated the relationship between oral health and nutritional status in elderly patients with chronic or acute pathology. The method used was a prospective cross-sectional clinical survey of 115 elderly patients (160 years old; average age 66.2 years) from the Clinical Foundation of the Dental School of the University of Medicine and Pharmacy of Iasi. The conclusion is that lack of education, taking more than 3 medications a day, physical inability to buy food or prepare meals, and difficulty in eating hard food are all closely related to malnutrition [6]. Although the analysis process is good, there are some problems in the research of certain theories.

RETRACTED

### 1.4. Innovation

The innovation of this article is (1) first of all, the innovation of the topic selection angle. This article is a new perspective from the perspective of topic selection. At present, there are not many researches that integrate medical image recognition, volleyball, nutritional food, athletes, and physical health. It is of exploratory significance. (2) The second is the innovation of methods. This paper combines medical image recognition technology with athlete diet research. (3) The third is the innovation of the experiment. This study has a certain reference value for athletes and sports lovers in other events and can help them adjust their diet.

## 2. Important Technology of Medical Image Recognition

### 2.1. Image Sampling

The discretization of the image in position [7] is called sampling, and the method is to uniformly sample the original image according to a square or regular hexagonal grid lattice.

Suppose two-dimensional continuous image, *I*(*a*, *b*), *a*, *b* ∈ (−∞, +∞), are a function of limited bandwidth [8]. That is, the Fourier transform of *I*(*a*, *b*) is *I*(*v*, *m*), then,

(1) $$\begin{array}{c} I\left(v,b\right)=\left\{I\left(v,b\right),v\in \left[-R_{S},R_{S}\right]\right.,b\in \left[-D_{A},D_{A}\right]. \end{array}$$

In the formula, *R*_*S*_ and *D*_*A*_ are the bandwidths in the *s* and *a* directions, respectively. The method of uniform sampling is to multiply the original image with the two-dimensional discrete sampling function *c* (*a*, *b*). The expression of *c* (*a*, *b*) is

(2) $$\begin{array}{c} c\left(a,b\right)=\overset{+\infty }{\underset{j=-\infty }{\sum }}\overset{+\infty }{\underset{k=-\infty }{\sum }}\partial \left(v-g\Delta a,b-h\Delta m\right). \end{array}$$

Among them, Δ*a* and Δ*m*, respectively, represent the sampling interval in the *a* and *m* directions [9] (sampling period).

The sampling function after sampling *I*(*a*, *b*) is *I*_*s*_(*a*, *b*):

(3) $$\begin{array}{c} I_{s}\left(a,b\right)=I\left(a,b\right)s\left(a,b\right)=I\left(a,b\right)\overset{+\infty }{\underset{c=-\infty }{\sum }}\overset{+\infty }{\underset{b=-\infty }{\sum }}\partial \left(a-z\Delta a,y-m\Delta v\right), \end{array}$$

(4) $$\begin{array}{c} I\left(a,b\right)=\overset{+\infty }{\underset{c=-\infty }{\sum }}\overset{+\infty }{\underset{v=-\infty }{\sum }}I\left(a\Delta b,n\Delta m\right)\partial \left(a-z\Delta a,y-m\Delta v\right). \end{array}$$

In the formula, the continuous function *I*(*a*, *b*) is moved into the summation formula and becomes *I*(*a*Δ*b*, *n*Δ*m*), which means that the value is only taken at the sampling point (*a*Δ*b*, *n*Δ*m*). So according to the convolution theorem in the Fourier transform, the frequency domain relation [10] is obtained as

(5) $$\begin{array}{c} Q_{c}\left(a,b\right)=\frac{1}{3\pi^{2}}R\left(a,b\right)*N\left(a,b\right). \end{array}$$

In the formula, *N* (*a*, *b*) represents the Fourier transform of the sampling function *N* (*x*, *y*) as

(6) $$\begin{array}{c} N\left(a,b\right)=\frac{1}{\Delta s}\frac{1}{\Delta b}\overset{+\infty }{\underset{-\infty }{\sum }}\overset{+\infty }{\underset{-\infty }{\sum }}\ell \left(w-c\frac{1}{\Delta s},x-z\frac{1}{\Delta g}\right). \end{array}$$

Substituting formula (6) into formula (5), and expanding the convolution formula, we can get

(7) $$\begin{array}{c} W_{s}\left(a,b\right)=\frac{1}{\Delta s}\frac{1}{\Delta b}\overset{+\infty }{\underset{-\infty }{\sum }}\overset{+\infty }{\underset{-\infty }{\sum }}Q\left(\alpha ,\beta \right)\left(w-c\frac{1}{\Delta s}-\alpha ,x-z\frac{1}{\Delta g}-\beta \right). \end{array}$$

From the above analysis, it can be seen that if the period extension spectrum of the sampled image does not overlap with each other during each period, then, the original image spectrum *I*(*a*, *b*) can be taken out through a two-dimensional ideal low-pass filter [11], and then after the inverse Fourier transform, the original image *I*(*v*, *m*) can be obtained. The periodic extension spectrum of the sampled image refers to extending the spectrum of the signal to occupy a wide frequency band, and the spectrum usually takes the angular frequency as the abscissa and the amplitude of each harmonic or the amplitude of the virtual exponential function as the ordinate. The frequency response of an ideal low-pass filter is

(8) $$\begin{array}{c} W\left(a,b\right)=\left\{\begin{array}{c} 1,a\in \left[-R_{U},R_{U}\right],s\left[-R_{V},R_{V}\right],\\ 0. \end{array}\right. \end{array}$$

The conditions for the spectrum not to alias each other are

(9) $$\begin{array}{c} \left\{\begin{array}{c} \frac{1}{\Delta a}\geq 3R_{U}\\ \frac{1}{\Delta b}\geq 3R_{U} \end{array}\right.\text{which is}\left\{\begin{array}{c} \Delta a\leq \frac{1}{2R_{U}},\\ \Delta b\leq \frac{1}{2R_{U}}. \end{array}\right. \end{array}$$

If the above sampling conditions cannot be met, the frequency of the sampled signal will overlap, that is, the frequency component higher than half of the sampling frequency will be reconstructed into a signal lower than half of the sampling frequency. The distortion caused by this spectrum overlap is called aliasing, and the reconstructed signal is called the aliasing substitute of the original signal, because the two signals have the same sample value. Once aliasing occurs, it cannot be eliminated, and the original signal will never be truly reproduced.

RETRACTED

This is the two-dimensional sampling theorem [12]. After sampling, the original continuous image becomes a positionally discretized sampled image *I*_*s*_(*a*, *b*)⟶*I*_*s*_(*c*, *v*), where *c* and *v* are integers satisfying the following relationship:

(10) $$\begin{array}{c} \left\{\begin{array}{c} 0\leq b\leq B-1,\\ 0\leq c\leq C-1. \end{array}\right. \end{array}$$

Here, *B* and *C* represent the number of uniform sampling points in rows and columns, and (*b*, *c*) represents a sampling point, which is the so-called pixel. Image recognition desampling is shown in Figure 1.

### 2.2. Image Feature Extraction Method

The Gabor function is a Fourier transform window method proposed by Dr. Gabor in 1964 and can also be regarded as a band filter. The Gabor filter is not only insensitive to local illumination [13] and image contrast changes but also has strong signal resolution capabilities in the time domain and frequency domain. The filtering result describes the gray information in different directions of the image. It can effectively describe the useful feature information in the image, so it has been widely used in feature output. In this paper, a two-dimensional Gabor filter [14] is used to capture the texture features of the test film image. The usual Gabor function [15] has the form:

(11) $$\begin{array}{c} w\left(a,b\right)=\left(\frac{1}{3\pi \partial_{a}\partial_{b}}\right)\exp\left[-\frac{1}{3}\left(\frac{a^{2}}{\partial^{2}}+\frac{b^{2}}{\partial^{2}}\right)+3\pi asc\right]. \end{array}$$

According to formula (11), Gabor wavelet is actually a sine wave signal modulated by a two-dimensional Gaussian function, where *s* is the modulation frequency, and *∂*_*a*_, *∂*_*b*_ is the standard deviation of the Gaussian function in the horizontal and vertical directions, respectively.

The Fourier transformation of the Gabor function is

(12) $$\begin{array}{c} W\left(a,b\right)=\exp\left\{-\frac{1}{2}\left[\frac{{\left(a-s\right)}^{2}}{\partial_{v}^{3}}+\frac{b^{2}}{\partial_{v}^{3}}\right]\right\}. \end{array}$$

Taking the function *h*(*a*, *b*) as the reference function and performing a scale transformation and rotation transformation on it, a series of self-similar Gabor wavelet functions can be obtained.

(13) $$\begin{array}{c} g_{ab}\left(c,v\right)=d^{-b}g\left(\bar{c},\bar{v}\right). \end{array}$$

For a *W* × *T* image 1, the convolution of its discrete Gabor wavelet transform can be expressed by the following equation:

(14) $$\begin{array}{c} W_{ab}\left(n,m\right)=\underset{s}{\sum }\underset{v}{\sum }W\left(a-s,b-v\right){g_{ab}}^{*}\left(d,b\right). \end{array}$$

Among them, 1 is the conjugate complex number of function 2, and *d* and *b* are the template sizes of the filter. Then, the energy of the image after Gabor transformation can be expressed as

(15) $$\begin{array}{c} W\left(a,b\right)=\underset{a}{\sum }\underset{b}{\sum }\left|W_{ac}\left(a,b\right)\right|. \end{array}$$

However, we generally do not choose energy information as texture features because energy features will bring classification errors. Therefore, this paper chooses texture feature vector {*η*_∞_, *∂*_∞_} composed of *s*_*a*_ energy mean *η*_*ab*_ and standard deviation *α*_*ab*_ as the texture feature of the test strip image.

(16) $$\begin{array}{c} \eta_{ab}=\frac{Q\left(a,b\right)}{\text{RT}}, \end{array}$$

(17) $$\begin{array}{c} \eta_{ab}=\sqrt{\frac{\sum_{v}\sum_{n}{\left(\left|W_{vn}\left(a,b\right)\right|-Q_{sa}\right)}^{2}}{\text{RT}}}. \end{array}$$

Gabor transform can fully describe image texture information and is a better method for extracting image texture features. It is widely used in image classification, texture analysis and segmentation, image recognition, and other fields.

RETRACTED

### 2.3. Medical Image Edge Detection

Edge detection [16] is a detection technique based on the existence of a certain discontinuity (or breakthrough) in the gray (or texture) characteristics between the object and the background. The edge of an image is one of the key features that image segmentation relies on, and it is also an important basis for image literary analysis and image recognition. Commonly used edge detection operators include Sobel operator [17, 18], Canny operator [19], Roberts operator [20], and Laplacian-Gaussian operator [21] and other nonlinear operators. We use the original Canny algorithm to perform edge detection on the CT image, and the result is shown in Figure 2:

Using these operators to detect the edges of the image, the effect is not ideal. Especially when the image is more complex and contains rich details, some nonlinear operators involve directionality and anisotropy, and it is difficult to completely detect the edges of the image. Medical image edge detection is an essential work and preprocessing step in medical image processing. Its main task is to determine and extract the edge information of the image and make preparations for image analysis, target recognition, and image coding. Medical image edge detection, like edge detection algorithms in other fields, also pays attention to performance indicators such as the accuracy of the detection results, the robustness of the algorithm, the speed of operation, and the degree of human participation.

Here are several definitions commonly used in edge detection:

**Definition 1 .**

On the interval [*s*_*a*_, *s*_*a*+1_], the variation *T*_*a* + 1_−*T*_*a*_ of the function *T* = *f*(*a*) is called the first-order forward difference on *s*_*a*_, with *c* = *s*_*a*+1_ − *s*_*a*_ as the step length. Recorded as

(18) $$\begin{array}{c} \Delta T=T_{a+1}-T_{a}. \end{array}$$

**Definition 2 .**

In interval [*s*_*a*_, *s*_*a*+1_], the variation *T*_*a* + 1_−*T*_*a*_ of the function *T* = *f*(*a*) is called the first-order backward difference on *s*_*a*_ with *c* = *s*_*a*+1_ − *s*_*a*_ as the step length. Recorded as

(19) $$\begin{array}{c} \Delta T=T_{a}-T_{a+1}. \end{array}$$

**Definition 3 .**

RETRACTED

Suppose *T* = *h*(*a*, *b*, *c*) is defined in a certain area of point *B*_1_(*a*_1_, *b*_1_, *c*_1_), *k* is the ray starting from point *B*_1_, *B*(*a*, *b*, *c*) is any point in the *k* direction, and *u* represents the distance between *D* and *D*_1_. If the limit:

(20) $$\begin{array}{c} \underset{p⟶1+}{\lim}\frac{S\left(p\right)-S\left(p_{1}\right)}{p}=\underset{p⟶1+}{\lim}\frac{\Delta_{v}S}{p}. \end{array}$$

## 3. Research on the Diet Pattern of Volleyball Players

### 3.1. The Overall Framework and Research Objects of the Research

By consulting a large number of relevant literature, we found that the research methods of dietary habits are single, and the nutritional status of the body caused by dietary habits includes many factors, such as energy, food type, macronutrients [22], micronutrients0 [23], and minerals [24], analyzing them separately cannot get the complete picture of athlete's nutritional status, and extracting key information can get the core of athlete's nutritional status and better serve sports practice. Therefore, we have made new attempts in methods, with the purpose of providing new ideas and methods for sports nutrition research. The overall framework of the research is shown in Figure 3.

Select 200 volleyball players from a higher vocational school as experimental subjects and divide them into two groups. The basic situation of the two groups of players is shown in Table 1.

In charge of the subjects of this survey, from the perspective of age distribution, there are 97 female volleyball players aged 14-19, and 113 female volleyball players aged 20-21. The proportions occupied were 48.5% and 51.5%. From the perspective of the number of training per week, the majority of female volleyball players train 3-6 times a week, with a total of 147 people, accounting for 73.5% of the entire survey. The number of athletes who train 1-2 times per week is as many as 19 athletes. The number of athletes who train more than 6 times a week is 34, accounting for 17% of the entire survey. At the time of each training session, the number of athletes who trained for 1-3 hours was 158, and the number of athletes who trained for more than 3 hours was 32, accounting for 79% of the total number of people in the survey. In terms of the average monthly food consumption of athletes, there are 17 people in the group below 200 yuan, 67 people in the 200-300 yuan group, 99 in the 300-400 yuan group, and 17 in the athlete group above 400 yuan. Their proportions in the survey were 8.5%, 33.5%, 49.5%, and 8.5%.

In summary, the age of female volleyball players in this higher vocational school tends to be younger, and the number of training sessions per week is mostly 3-6 times. The percentage of training times three or more times a week accounts for 95% of the entire survey. From this, it can be seen that the entire female volleyball player's training time is long, intense, and consumes a lot of energy. From the perspective of training time, there are no training courses within one hour, and all training time is maintained at more than one hour. This is also in line with the standards of volleyball competitions. A high-level and high-intensity volleyball game can last about 2-3 hours. Therefore, the curriculum design of this high-level female volleyball player conforms to the rules of volleyball competition. The basic situation of the sample of athletes interviewed by this subject in terms of age, number of training times per week, time of each training session, and average monthly food consumption is shown in Figure 4.

RETRACTED

### 3.2. Research Content

#### 3.2.1. Research Methods

1. Weighing method

During the survey period, the weight of the various food ingredients in the dishes and staple foods before being put into the pan is required to be weighed every day, that is, the weight of the edible part of the food, and the amount of various ingredients in each serving is calculated according to the number of meals and then calculated according to the food composition table to calculate the nutrient content of each serving. We also weigh the cooked weight of the dishes after cooking to calculate the ratio of raw to cooked, weigh the weight of the dishes actually ingested by the subjects to calculate the raw weight of the various food ingredients they consume, and then press the food composition table to calculate the intake of various nutrients. Meals are in the same canteen every day, and the canteen provides the same recipes. In addition, we have not made any intervention in the food choices of athletes.

(2) Dietary review method

Inquire and register all food and beverages consumed during the hour except for three meals. Then, calculate the average daily consumption of various foods.

(3) Measurement method

The first is the detection of body composition: on the first day of the diet survey, the height, weight, and body composition of the outstanding athletes in Fujian Province were measured with an empty stomach. The measurement content included height, weight, body fat content, body fat percentage, lean body mass, body water, total content, obesity rate, basal metabolic rate, electrical impedance, protein, muscle, minerals, intracellular fluid, extracellular fluid, and body state. The test instrument is a DX-200 body composition analyzer. Then, there were the inspection of nutritional biochemical indicators: in the early morning of the diet survey, venous blood was drawn from athletes before breakfast, and blood routine, serum total protein, serum albumin, serum globulin, ferritin, and other indicators were tested. Among them, we used flow cytometry to detect blood routine [25] (SYSMEX2100XE, 5 classification), biuret method to detect total protein (Olympus AU2700, Japan), and bromocresol green to detect serum albumin [26] (Olympus AU2700, Japan), using immunochemiluminescence method to detect serum ferritin (Beckmen automatic immunochemiluminescence instrument, USA).

RETRACTED

#### 3.2.2. Experimental Grouping

The first group is the diet intervention group, and the second group is the diet-free group. The *T* test results show that the diet intervention group and the control group can.

The differences in the amount and nutrient intake, energy balance, body weight, and body fat percentage are not significant, that is, the initial conditions are the same. The athlete's diet pattern is shown in Figure 5.

### 3.3. Experimental Results

There is no obvious difference in the daily diet patterns of athletes, as shown in Figure 6.

The first stage: athlete's body composition, dietary structure, and energy balance survey.

Among all vitamins, only the intake of vitamin E reaches the recommended value. The intake of other vitamins is lower than the daily recommended standard for athletes, especially the water-soluble vitamins B1, B2, and C. The lack of mineral intake is due to the athletes' less intake of beans, fish, and dairy products. Because athletes eat less beans, fish, and dairy products. The amount of various minerals in the diet of female athletes did not reach the recommended value. The reason for the insufficient intake of vitamins may be because athletes consume less fruits, beans, whole grains, and other foods, as shown in Table 2:

The second stage: the influence of diet intervention on athletes' body composition and energy balance.

1. Energy intake and energy supply ratio of the three major nutrients intervention

The energy supply ratios of protein, carbohydrate, and fat in the female intervention group all reached the recommended standards, but the energy supply ratios of the three major nutrients in the male and female control groups were still unreasonable, as shown in Table 3.

(2) Changes in energy intake and energy supply ratio of the three major nutrients in the intervention group before and after intervention

The energy intake of the female intervention group increased slightly after the intervention than before the intervention, but the difference was not significant. At the same time, the protein and carbohydrate energy supply of the two groups after the intervention increased compared with that before the intervention, and the fat energy supply was lower than that after the intervention than before the intervention. The difference was extremely significant (*P* < 0.02), as shown in Table 4.

(3) Changes in energy balance before and after intervention

After the intervention, the energy intake and energy consumption of the female intervention group maintained a balance, which was significantly changed from the negative balance before the intervention (*P* < 0.1). It can be seen from the data in Table 5 that the energy balance of the control group was −157.2 ± 129.6 before the intervention and −168.2 ± 125.2 after the intervention, which has always been negative. It is concluded that the energy balance of the female control group is always in negative balance before and after the intervention, as shown in Table 5.

RETRACTED

## 4. Experimental Analysis

### 4.1. Nutrient Intake Mode and Characteristic Factors of Athletes

The main component diagrams of nutrients ingested by different items and the analysis of characteristic parameters in the nutrient intake model are shown in Figures 7 and 8.

In Figure 7, we do a PCA analysis (PCA refers to principal component analysis or principal component analysis. It is a statistical analysis method to master the main contradictions of things. It can analyze the main influencing factors from multiple things, reveal the essence of things, and simplify complex problems. Here, it is applied to the analysis of athletes' nutritional intake, mainly analyzing the types of nutrients consumed by athletes.) of the nutrients and different items taken by the athletes and automatically fit them to obtain three principal components. The three components are protein, iron, and fierce. And Figure 8 shows that the three-day nutrient intake of athletes cannot be distinguished in the space composed of three principal components, and athletes of different events are relatively concentrated on the OPLS-DA score chart, while athletes of the same event show a trend of clustering. It shows that the nutrient intake of athletes in different sports has its own characteristics. The analysis of the characteristic parameters in the OPLS-DA model of nutrient intake by athletes is shown in Figure 9.

By solving the data, the VIP score chart obtained from Figure 9, the results are that athletes in the same sports event will be concentrated in one area, indicating that athletes in different sports have certain differences in the intake of nutrients, but the same sports the nutrients that athletes take in have a certain stability. The results show that the scalar quantities of VIP > 1 are carbohydrates, potassium, magnesium, total energy, protein, vitamin B2, iron, manganese, lysine, and zinc in order, indicating that the important variables of athletes' diet patterns in different sports are carbohydrates, protein, quantitative nutrients and total energy, as well as some micronutrients and minerals (potassium, magnesium, vitamin B2, iron, manganese, zinc, etc.).

RETRACTED

### 4.2. Changes in Body Weight and Body Composition of Athletes in Each Group Intervention

In the second stage, we learned that within one month of the intervention, the energy expenditure of all athletes hardly changed. This is consistent with the actual observation that all athletes did not participate in any competition during the intervention and training period, but the amount is still very high. This shows that sports trainings are not the reason for the changes in the weight and body composition of the athletes in each group.

Since all athletes were in a state of negative energy balance before the prediction, the female control group athletes lost significantly after one month. In addition, the percentage of female athletes in the control group did not change significantly, indicating that both body weight and body fat are decreasing. This change may be related to the characteristics of female energy supply, but its mechanism needs further study. Due to the increase in energy expenditure in the intervention diet, during the intervention period, the energy intake and energy expenditure of the female athletes in the intervention group were in a balanced state. Therefore, the weight of the female athletes in the intervention group did not change significantly after the intervention. Although the energy expenditure of all athletes remained almost unchanged within one month after the intervention, the percentage of body fat of athletes in the female intervention team decreased significantly. The reduction in food and the increase in protein-rich foods made them gain weight and improved their body composition.

Comparing athletes from the same overall intervention group and control group, their initial conditions are similar, but the final change trends are different. By analyzing all factors that affect the overall intervention expectations, we believe that the main reason for this change is diet. It seems that a reasonable diet can improve the weight and body composition of athletes, bringing them closer to the ideal range. Ideal body weight and body composition can not only ensure that athletes participate in large-capacity, high-intensity training but also can adopt contractual weight loss measures to smoothly reduce the normal weight of the competition. After weight loss, physical condition, and various competitions, the level will not drop significantly, which is essential for athletes. In the experiment, the weight and body composition of the athletes in the intervention group tend to change under ideal conditions, while the diet structure of the control group is in an absurd state, which will inevitably reduce the athletes' muscle strength and ultimately affect their athletic ability. The experimental results showed that 44.8% of the body weight and 40.2% of the body fat of all athletes were within the ideal range before the intervention. After the intervention, the percentage of all individuals whose weight was close to a reasonable range reached 48.5%, and the percentage of body fat within the recommended maximum range reached 41.3%.

RETRACTED

### 4.3. Investigation and Eating Habits

From the perspective of the main nutritional supplement sequence of athletes during regular training, 98% of athletes believe that cereals and rice noodles are always the most important source of nutrition, meat is the most important nutrition after cereals, and sports believe that they are training it must not be meat before, otherwise, it would be no nutritional supplement. This is also a nutritional supplement misunderstanding of today's volleyball players, thinking that meat is equivalent. Dairy products and eggs are ranked third, vegetables are ranked fourth, and fruits are ranked fifth. Sugar, as the most important substance for human energy, is used by most athletes.

From the perspective of the amount of supplementary nutrients for athletes during regular training, it can be clearly seen that meat, cereals, fish, eggs, vegetables, fruits, beans, and milk occupy the main position of athletes' daily diet. From the table below, the intake of nutrients in the daily diet of female volleyball athletes in Hunan Province can clearly see that, except for edible oil, the intake of other types of food structure is lower than the standard intake established by the National Nutrition Association. Among them, the intake of milk only accounts for 50% of the recommended value of the National Nutrition Association. Even athletes consider the most important staple food ingredients to be insufficient, accounting for only 78.22% of the standard value. Other various food ingredients, meat, vegetables, fruits, and soybean products accounted for 69.2%, 86.67%, 72%, and 80% of the standard value. It can be seen that the intake of most of the dietary nutrients of female volleyball players is lower than 80% of the standard intake, and a large group of athletes lack nutrient intake. The intake of nutrients in the daily diet of athletes is shown in Figure 10.

RETRACTED

In summary, there are mainly the following four eating habits. The first is a high-energy diet, excessive intake of starch and meat substances; and the second is a low-protein diet, which ignores the supplementation of body protein and makes the body the ratio of amino acids is not balanced. The third is the evening snack mode, and the fourth is the mode of quenching thirst with carbonated drinks after exercise. These are unhealthy eating patterns, which not only fail to replenish energy loss after exercise but also have no corresponding effect on relieving physical fatigue and muscle fatigue.

## 5. Conclusions

With the improvement of people's living standards and quality of life, health and health care as an emerging industry has begun to flourish, and people have begun to pay attention to dietary nutrition issues to improve their physical fitness and quality of life. Athletes, as a special group, are role models and representatives of national physical fitness to a certain extent. Therefore, it is essential to study the nutritional diet of athletes. Volleyball has become one of the most popular sports due to its simple game rules and venue standards, so it is essential for volleyball players to formulate a reasonable and scientific nutritious diet. This article draws several conclusions through analysis. One is that athletes have their own dietary patterns, and the other is that athletes' amino acid intake is positively correlated with body mass index and is related to the percentage of body fat. There are also some shortcomings in this research. Each female volleyball player's body structure is different. The conclusions drawn in this article are only suitable for general volleyball players. Due to the research funding and the validity of the research data, this research is unable to develop a scientific and complete set of meal plan is also one of the areas where future research needs to be done.

## Figures and Tables

**Figure 1:** Image recognition and sampling.

**Figure 2:** The original Canny algorithm edge detection.

**Figure 3:** The overall framework of the study.

**Figure 4:** Distribution of basic information of female volleyball players.

**Figure 5:** Athlete's diet pattern.

**Figure 6:** PCA analysis of food types and nutrients consumed in three days.

**Figure 7:** Principal component diagram of ingested nutrient PCA.

**Figure 8:** Analysis of characteristic parameters in the nutrient intake model of athletes.

**Figure 9:** Analysis of characteristic parameters in the OPLS-DA model of nutrient intake by athletes.

**Figure 10:** The intake of nutrients in the daily rations of female volleyball players.

RETRACTED

**Table 1:** The basic situation of the two groups of players.

Name	Age	Height (cm)	Weight (kg)	Sport level
Dong∗∗	18	173	62	Master
Su∗∗	14	179	61	Master
Qin∗∗	21	178	60	First level
Liu∗∗	21	182	63	First level
Yu∗∗	16	175	60	First level
Zuo∗∗	20	178	61	First level
Wu∗∗	19	177	62	Level 2
Miao∗∗	18	182	63	Level 2
Guo∗∗	17	177	64	Level 2
...				
Yang∗∗	15	175	60	Master
Wang∗∗	21	174	61	Master
Xie∗∗	16	172	62	First level
Tian∗∗	19	176	63	First level
Long∗∗	18	178	65	First level
Zeng∗∗	14	179	62	First level
Liang∗∗	20	182	64	Level 2
Xie∗∗	21	180	63	Level 2
Ke∗∗	20	176	62	Level 2
...				

**Table 2:** Average daily intake of vitamins and minerals in the surveyed athletes.

Minerals	Athlete
Vitamin A (*μ*gRE/d)	332.0 ± 509.2
Vitamin B1 (mg/d)	0.75 ± 0.34
Vitamin B2 (mg/d)	0.88 ± 0.29
Vitamin C (mg/d)	52.6 ± 26.8
Vitamin E (mg*α*-TE/d)	29.0 ± 15.7
Calcium (mg/d)	479.5 ± 207.5
Iron (mg/d)	21.5 ± 8.2
Zinc (mg/d)	8.4 ± 3.5
Selenium (*μ*g/d)	44.9 ± 20.3

**Table 3:** Energy intake and energy supply ratio of the three major nutrients after intervention in each group.

	Number of samples (people)	Energy intake (kcal/d)	Protein energy supply ratio (%)	Carbohydrate energy supply ratio (%)	Fat energy ratio (%)
Female intervention group	112	2458.3 ± 163.9	22.3 ± 1.7	62.5 ± 1.6	19.2 ± 1.8
Female control group	88	2285.8 ± 275.9	15.0 ± 2.2	61.5 ± 2.6	27.8 ± 1.58

**Table 4:** Changes in energy and energy supply ratios of the three major nutrients before and after intervention in the female intervention group.

	Energy intake (kcal/d)	Protein energy supply ratio (%)	Carbohydrate energy supply ratio (%)	Fat energy supply ratio (%)
Before intervention	2325.1 ± 242.3	14.5 ± 2.6	59.6 ± 3.2	29.6 ± 2.1
After the intervention	2425.3 ± 162.3	22.5 ± 1.9∗∗	62.6 ± 1.8∗∗	18.2 ± 1.9∗∗

**Table 5:** Changes in the energy balance of each group before and after intervention.

	Number of samples (people)	Energy balance before intervention (energy intake-energy expenditure)	Energy balance after intervention (energy intake-energy expenditure)
Female intervention group	112	−158.2 ± 156.2	−19.6 ± 92.3∗
Female control group	88	−157.2 ± 129.6	−168.2 ± 125.2

## Data Availability

All the data used is given in the paper.
